# A data science based standardized Gini index as a Lorenz dominance preserving measure of the inequality of distributions

**DOI:** 10.1371/journal.pone.0181572

**Published:** 2017-08-10

**Authors:** Alfred Ultsch, Jörn Lötsch

**Affiliations:** 1 DataBionics Research Group, University of Marburg, Marburg, Germany; 2 Institute of Clinical Pharmacology, Goethe - University, Frankfurt am Main, Germany; 3 Fraunhofer Institute of Molecular Biology and Applied Ecology - Project Group Translational Medicine and Pharmacology (IME-TMP), Frankfurt am Main, Germany; Universita degli Studi del Piemonte Orientale Amedeo Avogadro, ITALY

## Abstract

The Gini index is a measure of the inequality of a distribution that can be derived from Lorenz curves. While commonly used in, e.g., economic research, it suffers from ambiguity via lack of Lorenz dominance preservation. Here, investigation of large sets of empirical distributions of incomes of the World’s countries over several years indicated firstly, that the Gini indices are centered on a value of 33.33% corresponding to the Gini index of the uniform distribution and secondly, that the Lorenz curves of these distributions are consistent with Lorenz curves of log-normal distributions. This can be employed to provide a Lorenz dominance preserving equivalent of the Gini index. Therefore, a modified measure based on log-normal approximation and standardization of Lorenz curves is proposed. The so-called *UGini* index provides a meaningful and intuitive standardization on the uniform distribution as this characterizes societies that provide equal chances. The novel *UGini* index preserves Lorenz dominance. Analysis of the probability density distributions of the *UGini* index of the World’s counties income data indicated multimodality in two independent data sets. Applying Bayesian statistics provided a data-based classification of the World’s countries’ income distributions. The *UGini* index can be re-transferred into the classical index to preserve comparability with previous research.

## Introduction

Computational data science is a rapidly growing multidisciplinary field that uses advanced computing capabilities to understand and solve complex problem processes and systems [1]. It is aimed for extracting knowledge from data from various fields of research. The present analysis applied contemporary data science methods to the Gini index or coefficient [2], which is a common measure derived from Lorenz curves [3] to analyze the inequality of distributions [4]. The Gini index is used in economic data analyses such as the world’s countries' income distributions [5, 6] and its consequences [7]. Comparative analysis of the world’s countries' income inequalities is an active research topic [8–12].

However, analyses often remain descriptive and display the distribution of inequalities for different countries as a histogram [13]. Often software-default bin widths are used for the histograms. This imposes an arbitrary classification on the inequalities among countries. An example of this arbitrary classification is shown in Fig 1. A frequent observation in economic data is an uneven distribution (inequality) of the income in a country [14]. The resulting Gini indices are located between its defined borders of 0%, which is taken when all items are distributed at the same frequency such as all people in a society have exactly the same income, and 100% for maximum inequality as in the case that all income of a country goes to one person. However, the Gini index as a comparative measure of the inequality of distributions suffers from ambiguity [15, 16]. The same Gini indices may be associated with different Lorenz curves lying above or below the other, i.e., dominate each other, which indicates societies with more or less inequal income distributions[17]. Hence, the classical Gini index is not Lorenz dominance preserving.

**Fig 1:** Raw Gini indices of the latest Gini indices for the countries as estimated by the World Bank based on income. **Top**: The histogram shows the distribution of the raw Gini indices. **Bottom**: World map with countries colored according to the color ramp used in the histogram, i.e., low Gini index values are shown in green, high Gini index values are shown in dark red. Empty (white) regions indicate either lack of information or information judged as of poor quality by the publisher. The Fig has been created using the R software package (version 3.4.0 for Linux; http://CRAN.R-project.org/ [18]). The world map was drawn using the “mapCountryData” function of the R package “rworldmap” (South A.; https://cran.r-project.org/package=rworldmap [36]).

Thus, the Gini index addresses the generally important problem of the statistical analysis of skewed distributions and is a common measure in economic research. Considering above-mentioned weaknesses, a Lorenz dominance preserving replacement may be desirable. Therefore, in the present analysis, contemporary data science methods were used to (i) establish a suitable basis to standardize a meaningful equivalent of the Gini index, (ii) to derive a Lorenz dominance preserving modified Gini index, and (iii) to establish an adequate data-based classification of the World’s countries with respect to the inequalities of income distributions.

## Methods

### Data sets

Gini indices and income distributions of the world’s countries were obtained from the World Bank primary collection of development indicators publicly available at http://data.worldbank.org/data-catalog/world-development-indicators (accessed on May 1^st^, 2017). The World Bank’s estimates had been compiled from officially-recognized international sources and based on primary household survey data obtained from government statistical agencies and World Bank country departments (http://iresearch.worldbank.org/PovcalNet/index.htm). For the present analysis, the “distribution of income or consumption” table was downloaded on May 1^st^, 2017 from http://wdi.worldbank.org/table/2.9. It provided the World Bank’s estimates of the Gini index and the percentiles of the income distributions of n = 177 countries. Cases were acquired between the years 1995 and 2014 with a median year of acquisition of 2012 and an interquartile range of 2009–2014. Only data based on income and with the variable “Quality” indicating “average” or “high” quality were taken. The percentiles of the income distributions were translated into Lorenz curves using spline interpolation for all percentiles in the unit interval.

For replication of key findings, a second data set was obtained from the United Nations University World Institute for Development Economics Research at https://www.wider.unu.edu/download/WIID3.3 (accessed on October 20, 2016). This data set comprised the Gini indices and income distribution percentiles of n = 159 countries, with earliest measurements taken from 1867, however, most data were available for the period after 1960. To avoid dominance of well-documented countries, only the most recent 25 years were considered. Only data based on income and of “average” or “high” quality according to the variable “Quality” were taken. Following elimination of data also present in the World Bank’s data set, the second data set comprised n = 1,909 Gini indices and Lorenz curves of n = 149 countries with a median year of acquisition of 1990 (interquartile range 1972–1998). Again, the percentiles of the income distributions were used to calculate the corresponding Lorenz curves using spline interpolation.

### Data analysis

Data were analyzed using the R software package (version 3.4.0 for Linux; http://CRAN.R-project.org/ [18]) on an Intel Xeon^®^ computer running on Ubuntu Linux 16.04.2. The data science methods applied on the Gini indices followed three principal steps. **Firstly**, the empirical distribution of Gini indices was explored by analyzing their probability density function. This identified a concentration on a Gini index of 33.33% corresponding to the Gini index of the uniform distribution. Specifically, In general, the Gini index for a distribution that is uniform in the interval [a,b] deviates less than 5% from 33.33% if b ≥ 50 · a, which is assumed to hold for empirical income distributions. The uniform distribution and therefore, a Gini index of 33.33%, was taken as a realistic null hypothesis on the following basis. The “uniform” distribution is defined as a distribution where a finite number of values are equally likely to be observed. Thus, it is an inequality distribution as every member of, e.g., a population, has the same chance to earn, e.g., 1 dollar or 1,000,000 dollars. By contrast, the identity distribution is the distribution where every member of a population earns exactly the same amount. The Gini index for the identity distribution is 0%. Considering the implication of equal chances in just societies, the uniform distribution was considered to provide a standardization basis of the Gini index, whereas using the identity distribution would have provided a reference to an unrealistic setting where every member of a society earns the same amount of money.

**Secondly**, the ambiguity of the Gini index was addressed by approximating an equivalent log-normal Lorenz curve to the World’s countries’ income distributions. The standard deviation, *LN(S)* was identified as a parameter uniquely determining the associated Lorenz curve *L(S)*, serving as suitable approach at a modified Gini index that preserved Lorenz dominance. **Thirdly**, the distribution of that index was analyzed using a Gaussian mixture model. This allowed the application of Bayesian statistics for the calculation of a data-based classification of the World’s countries’ inequalities in income distributions.

#### Analysis of the empirical distribution of raw Gini indices

The probability density function of the Gini indices was analyzed using the Pareto density estimation (PDE), which is a kernel density estimator particularly suitable for the discovery of groups in data [19]. PDE analysis indicated a concentration of the probability density function on a Gini coefficient of 33.33% (Fig 2, dashed magenta lines). This seemed to be a consistent finding across the literature (see Fig 1 in [13], Fig 3 in [20], Fig 2 in [21], or Fig 3 in [22]). The observed center of the distribution corresponds to the Gini coefficient G_U_ = 1/3 = 33.33% of any uniform distribution *Uniform[0…m]*, *m > 0* [23]. A uniform distribution is characteristic for societies where all members have an equal chance to earn an income of any height. This suggested standardizing the Gini index to a measure that reflects its deviation from the uniform distribution. In contrast to the uniform distribution, the identity distribution, where all members of a society have the same income, has a Gini Index of 0%.

**Fig 2:** Comparative display of the probability density function of the distribution of raw Gini indices (**top**) and the novel UGini indices (**bottom**). The blue lines indicate the estimate by applying the Pareto Density Estimation (PDE) [19]. The dotted perpendicular magenta lines are drawn at the Gini coefficient of the uniform distribution at Gini = 33.33%, or at the UGini coefficient of the uniform distribution at UGini = 0%, which both intersected the PDEs at their maximum or very close to it. **Left**: Indices of countries estimated by the World Bank based on income. **Right**: Indices of countries of the test data set derived from the information provided by the United Nations University World Institute for Development Economics https://www.wider.unu.edu/download/WIID3.3. The differences in the distributions may be attributed to the different origins of the data sets or result from different methods in preprocessing (cleaning) of the data before publication. The Fig has been created using the R software package (version 3.4.0 for Linux; http://CRAN.R-project.org/ [18]).

#### Establishment of a Lorenz dominance preserving equivalent Gini index

Let *pdf(x)* denote the probability density function of a continuous random variable, *cdf(x)* denote the corresponding cumulative distribution function with inverse x(F), then the Lorenz curve for the distribution *L(x)* is defined by $L\left(x\right)=\frac{1}{m}\int_{-\infty }^{x}\left(x\;pdf\left(x\right)\right)$, where *m* = *∫ x* * *pdf* (*x*) *dx* denotes the mean of the distribution [23]. The Gini coefficient is then defined as *G* = 1 − 2 *∫L*(*x*) *dx* [23]. For a log-normal distribution $LogNorm\left(x,m,s\right)=\frac{1}{s\sqrt{2\pi }}\text{exp}\left(-\frac{{\left(\text{ln}\left(x\right)-m\right)}^{2}}{s^{2}}\right)$ the Lorenz curve is given as *LN* (*s*) = *erf* (*erf*^−1^ (*p*) − *s*) and its Gini coefficient as $2\text{erf}\left(\frac{S}{\sqrt{2}}\right)-1$ [14].

If a Gini index *G*_*1*_ of a distribution with Lorenz curve *L*_*1*_ is larger than a Gini index *G*_*2*_ of a distribution with Lorenz curve *L*_*2*_, then Lorenz curve *L*_*1*_ is not necessarily dominated by *L*_*2*_, i.e., does not necessarily lie completely below it (Fig 3). Hence, the Gini index is an ambiguous measure of the inequality of the underlying distribution. To address the problem of lacking Lorenz dominance of the classical Gini index, each empirical Lorenz curve was approximated by a by the Lorenz curve of a log-normal distribution, *LN(S)* called in the following “*equivalent log-normal Lorenz curve*”. This was obtained by fitting *LN(S)* to the empirical Lorenz curves by minimizing the mean sum of squared errors.

**Fig 3:** Lorenz curves describing different inequalities while delivering the same Gini index. Up to about 70% of the population the Lorenz curve indicated for Germany in 1960 a more inequal income distribution than for Costa Rica in year 1991. However, both curves possess the same Gini index of 48.4%. This illustrates the ambiguity from which the Gini index suffers. For comparison, the Lorenz curves of the uniform and identity distributions are displayed as green and black dashed lines, respectively. By contrast, the proposed UGini indices are UGini = 40.4 for Germany, and UGini = 40.0 for Costa Rica, hence, the ambiguity was solved in the novel index. The Fig has been created using the R software package (version 3.4.0 for Linux; http://CRAN.R-project.org/ [18]).

In the *equivalent log-normal Lorenz curve*, inequality depends on a single parameter, *S*, describing the dispersion of the log-normal distribution *LN(S)*, which uniquely determined the shape of the corresponding Lorenz curves *L(S)*. Therefore, *S* preserves Lorenz dominance and is robust against the *ambiguity of the original Gini index*. That is, if *S*_*1*_ *> S*_*2*_ holds for two log-normal distributions *LN(S*_*1*_*)* and *LN(S*_*2*_*)* it follows that Lorenz curve of *S*_*1*_ is nowhere above the Lorenz curve of *S*_*2*_, i.e., the distribution *LN(S*_*1*_*)* possesses more inequality than *LN(S*_*2*_*)* everywhere in the population. The observation of the concentration of the Gini indices on *G*_*u*_ = 33.33% suggested standardizing *S* to obtain a measure that reflects its deviation from the uniform distribution. The standardized form of this index was obtained as $UGini=\frac{S-S_{U}}{Mean\left(S,S_{U}\right)}$, where *S*_*u*_ = 0.6091 is the standard deviation of the log-normal distribution with Gini index *G*_*u*_. The agreement of the new inequality measure *UGini* with the raw Gini index was assessed by means of regression and correlation analysis (Pearson’s *r* [24]).

#### Modeling the multimodal distribution of the Gini indices

The PDE of *UGini* (see above subchapter) suggested a multimodal distribution, which was analyzed by fitting using a Gaussian mixture model (GMM) to the data as given by the equation $p\left(x\right)=\Sigma_{i=0}^{M}w_{i}N(x|m_{i},s_{i}),=\Sigma_{i=1}^{M}w_{i}\cdot \frac{1}{\sqrt{2\cdot \pi \cdot s_{i}}}\cdot e^{-\frac{{\left(x\;-\;m_{i}\right)}^{2}}{2\cdot s_{i}^{2}}}$, where *N*(*x*|*m*_*i*_, *s*_*i*_) denotes Gaussian probability densities (component, mode) with the parameters mean, *m*_*i*_, and standard deviation, *s*_*i*_ whereas the parameter *w*_*i*_ defines the relative contribution or weight (prior probability of the class) of each of the component Gaussians to the overall distribution adding up to a value of 1. The parameter *M* denotes the number of Gaussian components. GMM fitting was performed with the R package “AdaptGauss” (https://cran.r-project.org/package=AdaptGauss [25]). This interactive tool allows to visually adjust the fit, i.e., the numerical values could be optimized interactively with the root mean square error between empirical distribution (PDE) and GMM as the fit criterion. GMM optimization was done for up to seven components and the final model was selected on the basis of visual inspection of the fit, the Akaike information criterion [26], the statistical significance of a χ^2^ test estimating the likelihood that the final model did not adequately describe the data, and a quantile-quantile (QQ) plots. Replication of key results was addressed in the independent UN data set.

## Results

Gini indices in the World Bank’s data set varied between values of 24.3 and 63.7% (Fig 1). A maximum of the probability density function was observed close to a Gini index of 33% (Fig 2 top left, dotted magenta line) corresponding to the Gini index of the uniform distribution. This suggested a suitable basis for a standardized Gini index.

The ambiguity of the Gini index was addressed by approximating an equivalent log-normal Lorenz curve to the World’s countries’ income distributions. The *equivalent log-normal Lorenz curves*, *LN(S)*, provided a satisfactory fit of the Lorenz curves as indicated by low mean sums of squared errors with a mean of less than 0.5% and a maximum not exceeding 5%. From standardizing *S*, being a Lorenz dominance preserving descriptor of the inequality of a distribution described by a Lorenz curve, to the value of *S*_*u*_ = 0.6091 of the uniform distribution, the unambiguous standardized Gini index *UGini* was obtained.

As desired, the *UGini* was highly correlated with the log of the raw Gini indices (Pearson’s *r* = 0.9917, df = 152, p < 2.2 · 10^−16^). It was easily back-transferable into the raw Gini indices using *Gini* = *e*^0.009 ⋅ *UGini*+3.506^ where the y-intercept = 3.502 corresponds the log of 33.33% and reflects the centering of *UGini* on the uniform distribution and 0.009 is the proportionality factor between the indices scaled in percent (Fig 4). A jitter between the original and the back calculated indices (Fig 4 right panel) owes to the different treatments of Lorenz dominance by *UGini* as compared to the original Gini index. Hence, *UGini* was a valid alternative to the standard Gini index. The comparative shapes of the distributions of the original *Gini* indices and the novel *UGini* indices are shown in Fig 2 bottom.

**Fig 4:** Correlation dot plots between different variants of the Gini index analyzed in this paper. **Left**: Correlation between the unambiguous standardized Gini index obtained as $UGini=\frac{S-S_{U}}{Mean\left(S,S_{U}\right)}$, where *S*_*u*_ = 0.6091 denotes the standard deviation of the log-normal distribution with Gini index *G*_*u*_. and the log of the raw Gini indices. **Right**: Agreement of the original raw Gini index and the Gini index resulting from back transformation of the *UGini* parameter. The Fig has been created using the R software package (version 3.4.0 for Linux; http://CRAN.R-project.org/ [18]).

The probability density function of the parameter *UGini* was analyzed using a Gaussian mixture model. This provided an appropriate fit of the data when using a number of *M* = 4 Gaussians (Fig 5) based on the lowest Akaike information criterion for M = 1,…,7 modes (AIC = 7105.8, 7092.8, 7094.1, 7086.2, 7088.4, 7116.6 and 7100.2, respectively) and likelihood ratio tests that indicated improvement of the fits up until four modes bot not further). The obtained model (Table 1) described the distribution of the set of standardized Gini indices at a high significance level as supported by p < 10^−4^ in a χ^2^ test that indicated the probability that the model did not describe the data distribution. This was supported by visual inspection of the fit and a QQ plot (Fig 5 top right).

**Table 1:** Results of the Gaussian mixture modeling (GMM) given as $p\left(x\right)=\Sigma_{i=0}^{M}w_{i}N(x|m_{i},s_{i})$, where *m*_*i*_, *s*_*i*_ and *w*_*i*_ are the parameters mean, standard deviation and relative weight of each of the Gaussians, respectively, obtained for the *UGini* index data. The final model with an optimum number of *M* = 4 mixes was selected on the basis of the Akaike information criterion [26], visual inspection of the fit, the statistical significance of an χ^2^ test estimating the likelihood that the final model did not adequately describe the data, and a quantile-quantile plot (Fig 5).

Parameter	Gaussian #1	Gaussian #2	Gaussian #3	Gaussian #4
Mean	-32.14	0	26.29	49.07
Standard deviation	10.23	14.06	17.94	11.11
Weight	0.21	0.45	0.12	0.21
Bayes boundaries	-20.52	24.5	32.74	Inf

**Fig 5:** Distribution of the unambiguous standardized Gini indices (UGini) of countries as estimated by the World Bank based on income. **Top left**: The density distribution is presented as probability density function, estimated by means of the Pareto Density Estimation (PDE [19]; black line). A Gaussian mixture model (GMM) given as $p\left(x\right)=\Sigma_{i=0}^{M}w_{i}N(x|m_{i},s_{i})$, where *m*_*i*_, *s*_*i*_ and *w*_*i*_ are the parameters mean, standard deviation and relative weight of each of the Gaussians, respectively, was fit (red line) to the data, with a number of mixes of *M* = 4 (Gaussian, G #1 .. G #4) shown as differently colored lines. The Bayesian boundaries between the Gaussians are shown as perpendicular magenta-colored lines. **Top right**: A quantile-quantile plot comparing the observed distribution of standardized Gini indices with the distribution expected from the GMM (abscissa). **Bottom**: World map showing the countries classified for Gini index categories. The four categories correspond to the four Gaussian modes identified to best describe the distribution of the standardized Gini indices. The Gini index increases with the number of the category and low Gini index values are shown in green while high Gini index values are shown in dark red. Empty (white) regions indicate either lack of information or information judged as of poor quality by the publisher. The Fig has been created using the R software package (version 3.4.0 for Linux; http://CRAN.R-project.org/ [18]); specifically, the GMM was drawn using our R package “AdaptGauss” (https://cran.r-project.org/package=AdaptGauss [25]) and the world map was drawn using the “mapCountryData” function of the R package “rworldmap” (South A.; https://cran.r-project.org/package=rworldmap [36]).

Replication of the key findings in the Word Bank data set, i.e., of (i) the concentration of raw Gini indices on a value of 33.33% and (ii) the modal distribution of the indices suggesting a data-based classification of the World’s countries’ Gini indices was successful in the data set obtained from the United Nations University World Institute for Development Economics. Gini indices varied between values of 16.1 and 66.3% and displayed a maximum of the probability density function close to Gini = 33.33% (Fig 2 right, dotted magenta line). Again, a modal distribution of *UGini* was established with *M* = 4 components of the GMM, supported by the lowest value of the Akaike information criterion (AIC = 15893, 15668, 15623, 15619, 16627, 16622 and 16684 for 1,2,3,4,5,6,7 modes, respectively) and likelihood ratio tests again indicating significant improvements of the fits from 1 to 4 modes but not further improvement with 5 or more modes. The χ^2^ test with p < 10^−3^ indicated significance that the model described the data. A large Gaussian mode (class) contributing with a weight of *w*_*2*_ = 23% to the GMM (Gaussian #2, Fig 6) emerged again around an *UGini* value of zero.

**Fig 6:** Distribution of the unambiguous Gini indices of countries of the test data set derived from the information provided by the United Nations University World Institute for Development Economics https://www.wider.unu.edu/download/WIID3.3. **Left**: The density distribution is presented as probability density function, estimated by means of the Pareto Density Estimation (PDE [19]; black line). A Gaussian mixture model (GMM) given as $p\left(x\right)=\Sigma_{i=0}^{M}w_{i}N(x|m_{i},s_{i})$, where *m*_*i*_, *s*_*i*_ and *w*_*i*_ are the parameters mean, standard deviation and relative weight of each of the Gaussians, respectively, was fit (red line) to the data, with a number of mixes of *M* = 4 (Gaussian, G #1 .. G #4) shown as differently colored lines. The Bayesian boundaries between the Gaussians are shown as perpendicular magenta-colored lines. Empty (white) regions indicate either lack of information or information judged as of poor quality by the publisher. The Fig has been created using the R software package (version 3.4.0 for Linux; http://CRAN.R-project.org/ [18]); specifically, the GMM was drawn using our R package “AdaptGauss” (https://cran.r-project.org/package=AdaptGauss [25]). **Right**: A quantile-quantile plot comparing the observed distribution of standardized Gini indices with the distribution expected from the GMM (abscissa).

## Discussion

Using a data science approach, the present analysis was successful in (i) establishing a suitable basis to standardize an intuitive equivalent of the Gini index, (ii) deriving a Lorenz dominance preserving modified Gini index, and (iii) establishing an adequate data-based classification of the World’s countries with respect to the inequalities of income distributions. It resulted in the proposal of a novel *UGini* index that uses the Gini index of the uniform distribution as a basis for a meaningful standardization for a comparative measure of income inequalities. The *UGini* index replaces the original index with the standard deviation of a suitable log-normal approximation of Lorenz curves, thereby resolving the ambiguity of the classical index while preserving its origin from the Lorenz curve [2, 3] as an established approach at the inequality of a distribution. In general, the identification of Lorenz dominance is regarded as a difficult problem as discussed, for example, in [27].

The **first** focus of the present analysis was establishing an intuitive standardization of the inequality measure of a distribution. A frequent observation with the original Gini index is the uneven distribution (inequality) of the income in a country given in a year [14]. Gini indices are located between 0% when all items are distributed at the same frequency and all people in an egalitarian society have exactly the same income and 100% when all income of a country goes to one person. Both scenarios, however, are highly unlikely among the world’s countries. Empirical observations of Gini indices suggested a concentration on the uniform distribution with Gini = 33.33%, which was observed in the present data sets and can also be seen in previous publications [13, 20–22]. Hence, taking the uniform distribution and, in turn, the value 1/3 for the Gini index as a realistic null hypothesis was, in addition to the causes specified in the method section, found to be supported by the empirical evidence taken from two different databases.

Among income distributions in a country, the uniform distribution characterizes a society where all members have the same chance to earn an income of any size. For a comparative measure of income inequalities, this appeared to be a suitable anchor point to develop a standardized Gini index. Indeed, a consistent observation in this analysis was a mode of the Gini index distribution at 33.33%. This suggests a tendency toward uniform distribution in a considerable fraction of countries. However, in contrast to the identity distribution as the standard reference point of the Gini index where all members of a society have exactly the same income, the uniform distribution allows for inequality. The richest person may earn more than the person with the least income; uniform distribution only requires that the chance to earn any amount of income is equal.

The standardization of the modified Gini index, in particular of *LN(S)*, used the relative difference to the respective parameter value of the uniform distribution. For non-logarithmic data, the relative difference between values *a* and *b* is given as $RelativeDifference\left(a,b\right)=\frac{b\;-\;a}{0.5\;\cdot \;\left(a\;+b\right)}$. It has been demonstrated that this relates to return rates $r=\frac{b-a}{a}$ and to logarithmic ratios $LogRatio\;=log\frac{b}{a}$ [28]. Furthermore, the resulting parameters have a symmetric positive and negative scale ranging from -2 to 2. This means that the proposed standardization of the indices provides an intuitive measure of deviations (relative or log ratio) of an index from the uniform distribution. A value of zero in the standardized parameter indicates the uniform distribution. Positive values point a tendency toward more inequality while negative values indicate a tendency toward more equality up to egalitarian societies with an identity distribution of wealth.

A **second** focus of the present analysis was amending the ambiguity of the classical Gini index. Despite the fact that the Gini coefficient has been judged as one of the most efficient measurements of income inequality in the world [29], it is known to suffer from several shortcomings. As a main weakness, its incapability of differentiating different kinds of inequalities has been highlighted [30]. Specifically, Lorenz curves may intersect with each other, reflecting differing patterns of income distributions, but they can nevertheless result in similar Gini coefficient values [30]. Moreover, an importance of preference ordering has been pointed out, such as the Lorenz dominance on a set of Lorenz curves as a basis for assessing the degree of inequality [31]. Among proposed solutions to address the sensitivity of the Gini index to inequalities in the middle of the income distribution [30], the Atkinson index [32] incorporates an additional sensitivity parameter. The higher the value of this parameter, the more sensitive the Atkinson index becomes to inequalities at the bottom of the income distribution. Alternatively, the Generalized Entropy index [33] also uses a sensitivity parameter that allows to adjust how much inequalities at the top of the income distribution are reflected by this index.

In the present work, following replacement of the original index with the standard deviation of a suitable log-normal approximation of Lorenz curves, the novel *UGini* index solved the ambiguity of the original index while preserving the origin of the inequality measure from the Lorenz curve [2, 3] as an established approach to the inequality of a distribution. The choice of the log-normal distribution is in line with early proposals dated back in 1957 when the suitability of log-normal distributions for income distributions was presented [34]. Moreover, from an extensive comparison of several different distributions proposed as models for empirical income data, such as including gamma and beta types of distributions and others [35], the lognormal distribution was found to surpass the usage of other distributions in many practical applications (see from page 126). More recently, statistical testing of 15 different income distributions in Ghana, Africa, showed no significant deviation from log-normal distributions [29], which agrees with the present results of curve fitting. Of note, the present approach to analyze the distributions of Gini indices can be transferred easily to the above-mentioned indices.

A **third** focus of the present analysis was to make the measure of income inequality accessible to a data based classification to improve current, mainly descriptive, judgments of the World’s countries income distributions. The novel *UGini* measure of income equalities was accessible to the establishment of a data-driven classification of the world’s countries for income inequality that exceeds the arbitrary classification frequently used in presentations of Gini indices (Fig 1). Mathematical modeling of the distribution of *UGini* allowed obtaining precisely calculated limits from which a data based classification of the world’s countries in a given data set of income inequality could be derived (Fig 5). The present analysis shows that a detailed investigation of the probability density function of the Gini indices resulted in the observation that a third or more of the Gini indices are distributed around a mean of 33.33% that corresponds to the Gini Index of a uniform distribution. The analysis further hinted at a typical pattern of Gini indices. The fraction of countries that realize such a fair income distribution was found to be considerably large as this formed the main ode of the distributions (Fig 2). However, 10–40% of the countries, depending on the World Bank or United Nations origin of the data indicate a more homogenous income than resulting from fair chances, whereas more unfair conditions are common in almost half of the world’s countries.

## Conclusions

An unambiguous standardized equivalent of the Gini index is proposed as a novel measure of inequality in a distribution of data. The so-called *UGini* index was derived from data science driven analysis of the probability distribution of observed Gini indices of the world’s countries. Based on valid Lorenz curve approximation with a log-normal model of income distributions, the *UGini* index is highly correlated with the original raw Gini index while being Lorenz dominance preserving. Due to this high correlation, via *Gini* = *e*^0.009 ⋅ *UGini*+3.502^ the *UGini* index, scaled in percent, is easily re-transferable into the classical Gini index and therefore preserves comparability of analytical results with previous research. However, by centering its scale on the uniform distribution agreeing with the theory of a just society with respect to income distribution, the *UGini* index can be interpreted intuitively with respect to the justness of a society. Positive *UGini* indices measure the concentration of the income distributions onto an increasingly smaller fraction of the population (the richest). Negative *UGini* indices start with equivalent opportunities (uniform distribution) and measure the evenness of the distribution down to distribution where all individuals earn the same amount. Furthermore, the *UGini* index allows a precise data-adequate and reproducible classification with respect to income inequality based on Bayesian statistics. Thus, a novel measure of inequality is purposed that correlates with the original *Gini* index while correcting its Lorenz dominance weakness and rescaling it toward an intuitive measure of the justness of income distribution.
